The article "Early Sexual Debut among Ghanaian Women: Correlates and Psychological Effect" was published in 2021. Journal: Biomed Res Int.

# Early Sexual Debut among Ghanaian Women: Correlates and Psychological Effect

**DOI:** 10.1155/2021/5838510

**Published:** 2021-09-14

**Authors:** Abdul Rauf Alhassan, Kasim Abdulai, Mohammed Awal Alhassan

**Affiliations:** ^1^Department of Surgery, Tamale Teaching Hospital, P.O. Box TL 16, Tamale, Ghana; ^2^Department of Clinical Nutrition and Dietetics, School of Allied Health Sciences, University of Cape Coast, Ghana; ^3^Department of Obstetrics and Gynaecology, Tamale Teaching Hospital, P.O. Box TL 16, Tamale, Ghana

## Abstract

Early sexual initiation is linked to an increased risk of HIV/AIDS and other STIs among teenagers, as well as having multiple partners, not using contraception, unintended pregnancy, and illegal abortions. *Aim*. To identify the correlates and psychological effects of early sexual debut among not-in-union women in Ghana. A descriptive cross-sectional survey was used for this study using data from Ghana Multiple Indicator Cluster Survey (MICS) for the year 2017/2018. SPSS software was used for data analysis, bivariate analysis for association was done using chi-square, and the prediction was done using a binary logistic regression model. The national prevalence of nonmarital early sexual initiation this current study recorded was 56.9%. Predictors variables were age, 15-24/≥35 years (AOR = 1.51, 1.28-1.78), ever educated (AOR = 0.50, 0.43-0.60), urban address (AOR = 0.85, 0.74-0.98), married/single (AOR = 1.23, 1.07-1.42), cohabitation/single (AOR = 1.43, 1.19-1.72), Greater Accra Region/Upper West Region (AOR = 0.67, 0.49-0.92), and health insurance (AOR = 0.89, 0.79-0.998). As the wealth indices of the woman decrease from the richest to poorest, the likelihood of early sexual debut inversely increases: fourth/richest (AOR = 1.23, 1.04-1.45), middle/richest (AOR = 1.31, 1.09-1.58), second/richest (AOR = 1.38, 1.11-1.72), and poorest/richest (AOR = 1.44, 1.12-1.86); use of the internet (AOR = 0.58, 0.50-068); substance use and alcohol ever use (AOR = 1.32, 1.17-1.49); cigarette ever use (AOR = 2.58, 1.44-4.64); contraceptive use (AOR = 1.31, 1.16-1.49); and ever heard of HIV (AOR = 59, 0.42-0.82). In conclusion, the prevalence of early sexual debut is still high in Ghana, especially among the northern regions. Several factors predicted early sex debut, and low life satisfaction and happiness were related to early sexual debut.

## 1. Introduction

Sub-Saharan African youth continue to be a high-risk population for sexually transmitted infections (STIs), such as HIV/AIDS [1–3]. As a result, it is critical to prioritize this population's sexual and reproductive health, as they are the “window of hope” in the battle against the HIV/AIDS epidemic [2, 4]. This awareness has informed policies aimed at shielding young people from new infections through behavioral improvement initiatives in some nations, such as Ghana [1–3]. Early sexual initiation is also one of those focused behavioral modification areas.

The article "Early Sexual Debut among Ghanaian Women: Correlates and Psychological Effect" was published in 2021. Journal: Biomed Res Int.

The term “early sexual debut” commonly refers to having first sexual encounter before the age of 14 [5]. However, some works of literature have that early sexual initiation is sexual encounters that begin before the age of eighteen [6, 7]. Early sex initiation is often regarded as a risky sexual practice due to its negative consequences [6, 7]. In other words, early sexual initiation is linked to an increased risk of HIV/AIDS and other STIs among teenagers, as well as having multiple partners, not using contraception, unintended pregnancy, and illegal abortions [8]. Early sexual practice at a young age is a public health problem that is now widespread around the world, especially in developing countries [9]. Even though the age at sexual debut varies by location and by person, early adolescent sexual activity continues to be a problem with negative psychosocial and health consequences [10, 11].

One of the big predisposing factors that put youth at risk of HIV/AIDS is an early sexual start. Young people's sexual initiation exposes them to a slew of negative sexual and reproductive health consequences [12]. Young people who start having sex at a younger age are more likely than those who do not to have numerous and simultaneous sex partners, transactional sex, unsafe sexual activity, and contract STIs like HIV [12, 13]. Early sexual activity has also been linked to an increased risk of unintended pregnancies and poor academic performance, especially among school-aged children [14].

Early sexual debut is common in African settings, with rates ranging from 26.8% in Nigeria to 55 percent in Ghana [15, 16]. For adolescents to remain sexually abstinent, a dynamic interplay of variables such as sociocultural, faith, parent, and child connectedness plays a major role in the timing of sexual initiation [17, 18]. In Turi et al.'s study factors such as region, substance use (e.g., ever chewed khat, AOR = 2.02, 95% CI: 1.47, 2.77; ever drank alcohol, AOR = 1.83, 95% CI: 1.35, 2.48) and not knowing about family planning (AOR = 4.47, 95% CI: 2.22, 8.99) were found to have statistically important associations with early sexual debut in teenage females, whereas ever educational history decreases the odds of early sex initiation. An increase in wealth index from the poorest was associated with a decreased chance of early sexual initiation [19]. In another study, women's early sexual intercourse seems to be determined by substance use habits such as alcohol consumption, cigarette smoking, and khat chewing [6]. In a recent study community-level factors such as marriage, wealth, media exposure, and use of alcohol were influencers of early sexual debut in Ghana, Malawi, and Uganda [20].

The article "Early Sexual Debut among Ghanaian Women: Correlates and Psychological Effect" was published in 2021. Journal: Biomed Res Int.

Although various studies evaluating early initiation of sexual intercourse among youth have been conducted in Ghana, the majority of these studies are institution-based and concentrate on adolescents in school and university settings, except few such as that of Asante et al. [15]. Asante et al.'s study relied on data from the 2014 Ghana Demographic and Health Survey for sexually active youth aged 15 to 24, whereas this current study will rely on data from Ghana Multiple Indicator Cluster Surveys (MICS) sexually active women (15–49 years) focusing on nonmarital initial sexual activity. The study's main aim is to identify the correlates and psychological effects of early sexual debut among not-in-union women in Ghana.

## 2. Materials and Methods

A descriptive cross-sectional survey was conducted using data from the Ghana Multiple Indicator Cluster Survey (MICS) 2017/18. From October 2017 to January 2018, the Ghana Statistical Service surveyed with the assistance of partners such as the Ministry of Health; Ministry of Education; Ministry of Sanitation and Water Resources; Ministry of Gender, Children and Social Protection; Ghana Health Service; and Ghana Education Service. The United Nations Children's Fund (UNICEF) provided technical assistance, and the Statistics for Results Facility–Catalytic Fund provided financial support to UNICEF, KOICA, UNDP, USAID, and the World Bank (SRF-CF).

The sampling frame was the 2010 Ghanaian Population and Housing Census (PHC). All women between the ages of 15 and 49 who were either permanent residents or tourists who stayed in selected households the night before the survey (14609) were included.

### 2.1. Statistical Analysis

The findings were analyzed using SPSS version 20. (IBM Corp., 2011, NY). Tables with frequencies and percentages were used to explain the effects of categorical variables. The relationship between the dependent and independent variables was determined using the chi-square test. The predictor variables of early sexual initiation were identified using a binary logistic regression model. The statistical significance of the analysis was set at a *P* value of 0.05. The early sexual debut was done excluding those women who never had sexual intercourse and those with initial sexual activity from union (marriage or cohabitation).

### 2.2. Ethical Consideration

UNICEF's MICS team accepted the protocol for using the Ghana Multiple Indicator Cluster Survey 2017/18 dataset for this study. There was no need for ethical approval since this analysis required a secondary examination of a dataset without disclosing the participants' and their households' identities.

The article "Early Sexual Debut among Ghanaian Women: Correlates and Psychological Effect" was published in 2021. Journal: Biomed Res Int.

## 3. Results

### 3.1. Sociodemographic Characteristics of Study Participants

The majority of the study participants (40.6%) were between the ages of 15 and 24, and the majority (51.2%) were from rural areas. In terms of marriage, less than half of the respondents (43.5%) were married. More (13.8%) of the participants came from the Ashanti Region, with the Akan tribe accounting for 38.2% of the total. Health insurance coverage was only 56.7% among the study participants. A significant number (35.1%) of the women had a history of alcohol intake, about 92.9% of them ever heard of HIV/AIDS, and the majority (85.4%) had never used the internet. (Tables 1 and 2).

### 3.2. Prevalence of Early Sexual Initiation among Ghanaian Women

The national prevalence of nonmarital early sexual initiation this current study recorded was 56.9%, and in terms of regional prevalence, the highest (66.6%) prevalence was recorded in the Northern Region (now Northern, Savanna, and Northeast regions) and the lowest (39.7%) prevalence was recorded in the Greater Accra Region (Table 3). Chi-square analysis resulted in a significant relationship between early sexual debut and all independent factors included in this study (*P* < 0.005) (Tables 4 and 5).

### 3.3. Predictors of Early Sexual Debut among Study Participants

At the bivariate level of analysis, all independent variables were significantly associated with the early sexual debut and hence were further modeled using a binary logistic regression model to identify predictors of early sexual debut.  Table 6 presents estimates of the effects of selected predictors on the odds (Exp[*B*]) of reporting early sexual debut among the respondents.

The age of the woman at the time of the interview predicted history of early sex debut. Women of the age group 15-24 years were 1.5 times more likely to have experienced early sexual debut as compared to women of the age group 35 years and above (AOR = 1.51, 95%, C.I. = 1.28-1.78).

Women with a history of education (ever attended school) were 0.5 times more likely to have experienced early sexual debut as compared with women with zero histories of education (AOR = 0.50, 95%, C.I. = 0.43-0.60). Women with residence in urban areas were 15% less likely to have engaged in early sexual debut as compared to those from rural areas (AOR = 0.85, 95%, C.I. = 0.74-0.98). At the time of the survey, women in union relationships (marriage or cohabitation) predicted a history of early sexual debut. Those married were likely about 1.2 times to have experienced early child debut as compared to those who were single (AOR = 1.23, 95%, C.I. = 1.07-1.42). Also, those in cohabitation relationships were likely about 1.4 times to have experienced early sexual debut as compared to those women who were single (AOR = 1.43, 95%, C.I. = 1.19-1.72). From regional prediction, the early sexual debut was 33% less likely for women from the Greater Accra Region when compared to women from the Upper West Region (AOR = 0.67, 95%, C.I. = 0.49-0.92). In terms of health, women with health insurance were likely about 0.9 times to have experienced early sexual debut (AOR = 0.89, 95%, C.I. = 0.79-0.998). The economic status of the woman is implicated in the prediction of early sexual debut. As the wealth indices of the woman decreases from the richest to poorest, the likelihood of early sexual debut inversely increases: fourth/richest (AOR = 1.23, 95%, C.I. = 1.04-1.45), middle/richest (AOR = 1.31, 95%, C.I. = 1.09-1.58), second/richest (AOR = 1.38, 95%, C.I. = 1.11-1.72), and poorest/richest (AOR = 1.44, 95%, C.I. = 1.12-1.86). The use of the internet was a protective variable in the study as those with a history of internet use were 42% less likely to have engaged in early sexual debut (AOR = 0.58, 95%, C.I. = 0.50-068). History of substance use (alcohol and cigarettes) predicted early sexual debut. Those with alcohol ever use were 1.3 times more likely to have engaged in early sexual debut (AOR = 1.32, 95%, C.I. = 1.17-1.49), and those with cigarette ever use were 2.6 times more likely to have engaged in early sexual debut (AOR = 2.58, 95%, C.I. = 1.44-4.64). Those with a history of contraceptive use were 1.3 times more likely to have engaged in early sexual debut (AOR = 1.31, 95%, C.I. = 1.16-1.49). Women who ever heard of HIV were 41% less likely to have engaged in early sexual debut (AOR = 59, 95%, C.I. = 0.42-0.82).

The article "Early Sexual Debut among Ghanaian Women: Correlates and Psychological Effect" was published in 2021. Journal: Biomed Res Int.

### 3.4. The Psychological Effect of Early Sexual Debut

Participant life satisfaction was done using the score of the life satisfaction ladder step (numbered from 0 to 10), where 0 represented the lowest life satisfaction and 10 the highest level of satisfaction. Different levels of life satisfaction were specified based on recommendations from the HBSC protocol (http://www.hbsc.org), and similar papers: those with a low score of 0–6, were classified as unsatisfied, and those with an average score of 7–8 and high scores of 9–10 were classified as satisfied. And with the estimation of overall happiness, respondents were asked would you say you are (1) very happy, (2) somewhat happy, (3) neither happy nor unhappy, (4) somewhat unhappy, and (5) very unhappy? Those with responses of very happy and somewhat happy were classified as happy, and those with responses of neither happy nor unhappy, somewhat unhappy, and very unhappy were classified as unhappy.

This study further identified a significant relationship between overall life satisfaction and early sexual debut. Those without a history of the early sexual debut were more likely about 7% to be satisfied with life as compared to those with early sexual debut history (OR = 1.07, 95% C.I. 1.02-1.12). And in terms of overall life happiness, those without a history of the early sexual debut were more likely about 4% to be happy with life as compared to those with early sexual debut history (OR = 1.04, 95% C.I. 1.01-1.06) (Table 7).

## 4. Discussion

Early sexual debut is common in African settings, with rates ranging from 26.8% in Nigeria to 55 percent in Ghana [15, 16]. In this current study, the national prevalence of nonmarital early sexual initiation this current study recorded was 56.9% and in terms of regional prevalence, the highest (66.6%) prevalence was recorded in the Northern Region (now Northern, Savanna, and Northeast regions) and the lowest (39.7%) prevalence was recorded in the Greater Accra Region.

At the bivariate level of analysis, all independent variables were significantly associated with the early sexual debut and hence were further modeled using a binary logistic regression model to identify predictors of early sexual debut. The age of the woman at the time of the interview predicted history of early sex debut. Women of the age group 15-24 years were likely about 1.5 times to have experienced early sexual debut as compared to women of the age group 35 years and above. Also, in a similar study, the odds of earlier sexual debut history were higher among women of age group 15-19 years as compared to those above 19 years [15].

Also, women with a history of education (ever attended school) were only likely about 0.5 times to present with a history of early sexual debut as compared with women with zero history education. Similar to Asante et al.'s study, females with no formal education and those with only a basic education were more likely to make an early sexual debut [15]. Early sexual activity has also been linked to an increased risk of unintended pregnancies and poor academic performance, especially among school-aged children [14].

From regional prediction, the early sexual debut was 33% less likely for women from the Greater Accra Region when compared to women from the Upper West Region. Also, similar to Turi et al.'s study, region of the respondents was found to have statistically important associations with an early sexual debut [19]. And women residing in urban areas were 15% less likely to engage in early sexual debut as compared to those from rural areas, and this was confirmed by Asante et al.'s study that women in rural areas had chances of engaging in early sexual debut as compared to those from rural areas [15]. It has also been suggested that young adults from less-affluent backgrounds believe they have fewer opportunities in life and may lack the educational, job, and leisure motivator compared to those in urban areas [21, 22].

The article "Early Sexual Debut among Ghanaian Women: Correlates and Psychological Effect" was published in 2021. Journal: Biomed Res Int.

It is documented that females with access to modern contraceptives are more likely to engage in sexual activities, which may have affected earlier sexual debut activity. Also, in this present study, those with a history of contraceptive use were likely about 1.3 times to have engaged in early sexual debut, and women with health insurance were likely 0.9 times to engage in early sexual debut. Internet access is a source of entertainment and information, and in this study, use of the internet was a protective variable study as those with a history of internet use were 42% less likely to have engaged in early sexual debut. The risk of an early sexual debut is found to be increased when people had only limited access to the media, and this risk was found to be higher in rural areas [15].

In a recent multicenter study, community-level factors such as marriage were identified as an influencer of early sex debut in Ghana, Malawi, and Uganda [20]. And in this current study, at the time of the survey, women in union relationships (marriage or cohabitation) predicted history of early sexual debut. Those married were about 1.2 times more likely to have experienced early child debut as compared to those who were single. Also, those in cohabitation relationships were likely about 1.4 times to present the history of early sexual debut as compared to those women who were single. However, this study isolated early marriage as a factor of early sex debut.

Individuals who have their first sexual experience at a young age are more likely to participate in risky activities that put them at risk of contracting STIs or HIV. Early sexual debutants are more likely to have a history of STIs and have a higher risk profile, which includes having multiple sex partners, inconsistent condom usage, pay for sex, a history of sexual harassment, and teenage pregnancy [23]. Maybe, this explains the reason why in this present study, women who ever heard of HIV were 41% less likely to have engaged in early sexual debut.

The economic status of the woman is implicated in the prediction of early sexual debut. As the wealth indices of the woman decrease from the richest to poorest, the likelihood of early sexual debut inversely increases. This is in line with earlier studies which also found household rich wealth status as a protective factor for early sex debut in Ghana [12, 15].

The article "Early Sexual Debut among Ghanaian Women: Correlates and Psychological Effect" was published in 2021. Journal: Biomed Res Int.

History of substance use (alcohol and cigarette) predicted early sexual debut. Those with alcohol ever use were more likely about 1.3 times to engage in early sexual debut, and those with cigarette ever use were likely about 2.6 times to engage in early sexual debut. In another study, women's early sexual intercourse seems to be determined by substance use habits such as alcohol consumption, cigarette smoking, and khat chewing [6].

Early adolescent sexual activity continues to be a problem with negative psychosocial and health consequences [10, 11]. The strongest link is discovered in the youngest individuals, with depressed people nearly five times more likely than nondepressed individuals to have had intercourse [24]. And in this present study, in terms of overall life happiness, those without a history of the early sexual debut were more likely about 4% to be happy with life as compared to those with early sexual debut history. Also, this study further identified a significant relationship between overall life satisfaction and early sexual debut. Those without a history of the early sexual debut were more likely about 7% to be satisfied with life as compared to those with early sexual debut history. Negative emotional responses to first sexual encounters may also be influenced by psychological factors such as regret or a lack of readiness, which are more common in people who initiate sexual activity early than their on-time initiating peers [25].

Since the research relied on secondary data for interpretation, not all factors related to the subject were examined.

## 5. Conclusion

The prevalence of early sexual debut is still higher in Ghana, especially among the northern regions. Several factors predicted early sex debut, and low life satisfaction and happiness were related to early sexual debut. There is a need for policy enforcement to promote female education and reduce poverty.

## Figures and Tables

**Table 1:** Socioeconomic factors of the respondents.

		Frequency	Percentage
Age group	15-24 years	5836	40.6%
	25-34 years	3837	26.7%
	35 years and above	4701	32.7%
Ever attended school	Yes	11283	78.5%
	No	3091	21.5%
Area	Urban	7134	48.8%
	Rural	7475	51.2%
Marital status	Married	6246	43.5%
	Cohabitation	1655	11.5%
	Single	6473	45.0%
Region	Western	1350	9.2%
	Central	1319	9.0%
	Greater Accra	1830	12.5%
	Volta	1303	8.9%
	Eastern	1440	9.9%
	Ashanti	2022	13.8%
	Brong Ahafo	1323	9.1%
	Northern	1499	10.3%
	Upper East	1170	8.0%
	Upper West	1353	9.3%
Ethnicity	Akan	5577	38.2%
	GA/Dangme	1142	7.8%
	Ewe	1758	12.0%
	Guan	513	3.5%
	Gruma	600	4.1%
	Mole Dagbani	3212	22.0%
	Grusi	598	4.1%
	Mande	73	0.5%
	Other	1131	7.7%
Health insurance	With insurance	8152	56.7%
	Without insurance	6222	43.3%
Functional difficulties (age 18-49 years)	Has functional difficulty	1125	9.0%
	Has no functional difficulty	11403	91.0%
Wealth index quintile	Poorest	3383	23.5%
	Second	2412	16.8%
	Middle	2680	18.6%
	Fourth	2720	18.9%
	Richest	3179	22.1%

The article "Early Sexual Debut among Ghanaian Women: Correlates and Psychological Effect" was published in 2021. Journal: Biomed Res Int.

**Table 2:** Other exposure factors.

		Frequency	Percentage
Frequency of watching TV	Not at all	4623	32.2%
	Less than once a week	1473	10.2%
	At least once a week	2321	16.1%
	Almost every day	5957	41.4%
Ever used internet	Yes	2005	14.6%
	No	11713	85.4%
Ever taken alcohol	Yes	5040	35.1%
	No	9334	64.9%
Ever tried cigarette smoking	Yes	130	0.9%
	No	14244	99.1%
Ever used a contraceptive method to avoid pregnancy	Yes	2367	20.7%
	No	9079	79.3%
Ever circumcised	Yes	672	6.4%
	No	9787	93.6%
Ever heard of HIV or AIDS	Yes	13353	92.9%
	No	1020	7.1%

**Table 3:** Prevalence of nonmarital early sexual debut in Ghana among women.

		Early sexual debut			
		No		Yes	
Region	Western	457	41.4%	646	58.6%
	Central	463	43.2%	608	56.8%
	Greater Accra	866	60.3%	569	39.7%
	Volta	399	35.6%	722	64.4%
	Eastern	497	41.8%	691	58.2%
	Ashanti	790	49.7%	801	50.3%
	Brong Ahafo	472	43.7%	607	56.3%
	Northern	358	33.4%	713	66.6%
	Upper East	299	36.4%	522	63.6%
	Upper West	335	34.4%	638	65.6%
Total		4936	43.1%	6517	56.9%

**Table 4:** Chi-square association between socioeconomic factors and early sex debut.

		Early sexual debut		*X* ^2^	*P* value
		NO	YES		
Age group	15- 24 years	1230	2246	143.763	≤0.001
	25-34 years	1769	1813		
	35 years and above	1937	2458		
Ever attended school	Yes	4151	4606	281.032	≤0.001
	No	785	1911		
Area	Urban	2888	2638	365.675	≤0.001
	Rural	2048	3879		
Marital status	Married	2483	3318	30.666	≤0.001
	Cohabitation	613	1013		
	Single	1840	2186		
Region	Western	457	646	315.567	≤0.001
	Central	463	608		
	Greater Accra	866	569		
	Volta	399	722		
	Eastern	497	691		
	Ashanti	790	801		
	Brong Ahafo	472	607		
	Northern	358	713		
	Upper East	299	522		
	Upper West	335	638		
Ethnicity	Akan	2115	2429	112.867	≤0.001
	Ga/Dangme	458	475		
	Ewe	661	799		
	Guan	133	282		
	Gruma	144	324		
	Mole Dagbani	898	1406		
	Grusi	154	263		
	Mande	20	34		
	Other	351	504		
Health insurance	Yes	3016	3538	53.266	≤0.001
	No	1920	2979		
Functional difficulties (age 18-49 years)	Yes	402	597	9.316	0.002
	No	4534	5480		
Wealth index quintile	Poorest	760	1819	676.189	≤0.001
	Second	688	1310		
	Middle	874	1307		
	Fourth	1055	1157		
	Richest	1559	924		

**Table 5:** Chi-square association between other exposure factors and early sexual debut.

		Early sexual debut		*X* ^2^	*P* value
		No	Yes		
Frequency of watching TV	Not at all	1243	2383	212.409	≤0.001
	Less than once a week	461	670		
	At least once a week	765	993		
	Almost every day	2467	2471		
Ever used internet	Yes	967	597	305.442	≤0.001
	No	3615	5822		
Ever taken alcohol	Yes	1876	2657	8.972	0.003
	No	3060	3860		
Ever tried cigarette smoking	Yes	42	83	4.649	0.031
	No	4894	6434		
Ever used a method to avoid pregnancy	Yes	948	1312	7.097	0.008
	No	2882	3496		
Ever circumcised	Yes	166	387	64.823	≤0.001
	No	3701	4059		
Ever heard of HIV or AIDS	Yes	4745	5953	104.427	≤0.001
	No	191	564		

The article "Early Sexual Debut among Ghanaian Women: Correlates and Psychological Effect" was published in 2021. Journal: Biomed Res Int.

**Table 6:** Binary logistic regression for predictors of early sexual debut.

	*B*	Sig.	AOR	95% C.I. for AOR	
				Lower	Upper
≥35 years		0.000			
15-24 years	0.409	0.000	1.506	1.280	1.771
25-34 years	-0.045	0.523	0.956	0.834	1.097
Ever attended school (yes/no)	-0.686	0.000	0.503	0.426	0.595
Area (urban/rural)	-0.159	0.029	0.853	0.740	0.984
Single		0.000			
Married	0.209	0.003	1.232	1.072	1.416
Cohabitation	0.359	0.000	1.431	1.192	1.718
Upper West		0.001			
Western	0.083	0.603	1.087	0.794	1.487
Central	-0.007	0.968	0.993	0.716	1.378
Greater Accra	-0.398	0.012	0.672	0.492	0.916
Volta	0.196	0.295	1.217	0.843	1.757
Eastern	-0.082	0.619	0.921	0.666	1.274
Ashanti	-0.041	0.783	0.960	0.719	1.283
Brong Ahafo	-0.138	0.386	0.871	0.639	1.189
Northern	-0.060	0.680	0.942	0.708	1.253
Upper East	0.201	0.137	1.223	0.938	1.595
Other tribes		0.223			
Akan	0.038	0.748	1.039	0.822	1.314
GA/Dangme	-0.058	0.703	0.943	0.700	1.272
Ewe	-0.150	0.336	0.861	0.634	1.168
Guan	0.158	0.428	1.171	0.793	1.730
Gruma	0.258	0.186	1.294	0.883	1.895
Mole Dagbani	-0.147	0.254	0.863	0.671	1.111
Grusi	0.039	0.833	1.040	0.724	1.492
Mande	0.106	0.794	1.112	0.500	2.473
Health insurance (yes/no)	-0.118	0.046	0.889	0.792	0.998
Disability (yes/no)	0.046	0.648	1.047	0.860	1.275
Richest		0.022			
Poorest	0.367	0.005	1.443	1.117	1.863
Second	0.322	0.005	1.380	1.105	1.724
Middle	0.271	0.005	1.311	1.085	1.584
Fourth	0.204	0.017	1.227	1.038	1.450
Watch TV almost every day		0.490			
Not at all	-0.107	0.222	0.899	0.758	1.067
Less than once a week	-0.031	0.756	0.969	0.795	1.182
At least once a week	0.042	0.616	1.043	0.885	1.228
Ever used internet (yes/no)	-0.542	0.000	0.582	0.495	0.683
Alcohol ever use (yes/no)	0.278	0.000	1.320	1.173	1.486
Cigarette ever use (yes/no)	0.948	0.002	2.580	1.435	4.640
Ever use contraceptive (yes/no)	0.272	0.000	1.313	1.159	1.488
Done FGM (yes/no)	0.199	0.145	1.221	0.933	1.596
Ever heard of HIV (yes/no)	-0.531	0.002	0.588	0.419	0.824

**Table 7:** Early nonmarital sexual debut and overall life satisfaction and happiness.

		Overall life satisfaction		OR (C.I.)	*P* value
Satisfied	Not satisfied				
Early sexual debut	No	1899	3029		0.01
		38.5%	61.5%	1.07 (1.02-1.12)	
	Yes	2353	4153		
		36.2%	63.8%		
		Overall life happiness		OR (C.I.)	*P* value
Happy	Unhappy				
Early sexual debut	No	3750	1186		0.01
		76.0%	24.0%	1.04 (1.01-1.06)	
	Yes	4778	1739		
		73.3%	26.7%		

The article "Early Sexual Debut among Ghanaian Women: Correlates and Psychological Effect" was published in 2021. Journal: Biomed Res Int.

## Data Availability

All data related to the findings of this study are available from the Multiple Indicator Cluster Survey (MICS) website upon request.
